# SOX8 Knockdown Overcomes Enzalutamide Resistance in Castration-Resistant Prostate Cancer by Inhibiting the Notch Signaling Pathway

**DOI:** 10.1155/2022/9235837

**Published:** 2022-10-06

**Authors:** Zhongbo Du, Xiaobin Chen, Pingyu Zhu, Wei Sun, Qi Lv, Shulin Cheng, Xuesong Yang, Xiaodong Yu

**Affiliations:** ^1^Department of Clinical Medicine, North Sichuan Medical College, Nanchong, China; ^2^Department of Urology, Affiliated Hospital of North Sichuan Medical College, Nanchong, China; ^3^Department of Urology, Fuling Center Hospital of Chongqing, Chongqing, China; ^4^The First Affiliated Hospital of Chongqing Medical University, Chongqing, China; ^5^Department of Operation, Affiliated Hospital of North Sichuan Medical College, Nanchong, China

## Abstract

Castration-resistant prostate cancer (CRPC) is still challenging to treat. Dissatisfaction with androgen signal-targeted therapy forces people to look for other treatment strategies. Therefore, this study is aimed at exploring the role of SOX8/Notch signaling in CRPC. The upregulation of SOX8, Notch4, and Hes5 indicated a poor progression-free survival (PFS) in CRPC patients. The expression of these proteins was also upregulated in enzalutamide-resistant LNCaP cells (Enza-R). Moreover, knocking down SOX8 inhibited malignant biological behaviors and decreased the activation of Notch signaling in Enza-R cells. Importantly, knocking down SOX8 obviously reversed the enzalutamide resistance in Enza-R cells, while RO0429097 (a *γ* secretase inhibitor inactivates Notch signaling) exerted similar effects. At last, we found that both SOX8 knockdown and/or RO0429097 suppressed tumor growth and bone metastasis *in vivo*. Altogether, our study indicated that the SOX8/Notch signaling is involved in CRPC and that these enzymes are possible targets to develop novel treatment for CRPC.

## 1. Introduction

Prostate cancer (PCa) is the most common cancer among men and represents one of the leading causes of cancer-related deaths in developed countries [1]. For advanced PCa, androgen deprivation therapy (ADT) is the mainstream therapy. However, most patients with advanced PCa develop a castration-resistant prostate cancer (CRPC) within 18-24 months after ADT [2, 3]. Unfortunately, current treatment strategies, including endocrine therapy, such as abiraterone and enzalutamide, and chemotherapy, result in poor long-term survival for CRPC patients [4–8]. Therefore, other molecular mechanisms that lead to CRPC have been investigated as an attempt to uncover novel therapeutic targets.

The Notch signaling pathway is highly conserved in mammalian cells as it determines the fate and differentiation of cells. At the same time, it participates in the development of many organs, including the prostate [9, 10]. Interestingly, there is a controversy about whether the Notch signaling pathway acts as a tumor suppressor or as an oncogene [11–16]. Excessive activation of the Notch signaling pathway has been reported in PCa, including in patients with CRPC [17–19]. Overexpression of Notch signaling molecules has been associated with PCa, while downregulation of Notch receptors inhibited malignant biological behaviors of PCa cells [20–24]. More importantly, Notch inhibitors (*γ*-secretase inhibitors), such as PF-3084014 and GSI-IX, enhance the efficacy of ADT in PCa [25–27]. In addition, our recent study has indicated that PF-3084014 partly reverses enzalutamide resistance in CRPC cells by inhibiting the Notch1 receptor [28]. Chemoresistance in PCa has also been associated with the dysregulation of Notch2 receptors [29, 30]. Despite these studies, underlying mechanisms of Notch receptors involved in ADT resistance and CRPC are still unclear.

The SOX (SRY-related HMG-box) family of genes includes approximately 30 different subtypes, termed from A to H. These genes are found in multiple types of progenitor cells and play a key role in the regulation of cell development [31]. SOX8 belongs to SOX group E, and it was shown to be overexpressed in various cancer types including triple-negative breast cancer (TNBC), ovarian cancer, and tongue squamous cell carcinoma [32–34], while promoting the tumorigenesis and progression of tumors. Importantly, SOX8 was shown to be responsible for the chemotherapy resistance of multiple cancers [32, 34]. However, the role of SOX8 in PCa, especially in CRPC, is still unknown.

In this study, we reported that SOX8, Notch4, and Hes5 were significantly elevated in CRPC samples when compared with those of PCa samples. Increased levels of SOX8, Notch4, and Hes5 represented a worse prognosis for CRPC patients. We also found that these enzymes were upregulated in CRPC cells (named as Enza-R cells), when compared to their parental cells, LNCaP. Moreover, downregulating SOX8 significantly inhibited malignant behaviors of both CRPC and DU145 cells and reversed the resistance to enzalutamide by decreasing activities of Notch signaling. Importantly, a *γ*-secretase inhibitor (Notch signaling inhibitor) RO0429097 obviously restored the sensitivity of Enza-R cells to enzalutamide. Finally, SOX8 knockdown or RO0429097 was able to block the growth and bone metastasis of Enza-R cells *in vivo*. Taken together, our results indicate that the SOX8/Notch signaling axis may be a promising therapeutic strategy for CRPC.

## 2. Materials and Methods

### 2.1. Patients and Tissue Samples

A total of 45 PCa samples were collected from the Affiliated Hospital of North Sichuan Medical College, Nanchong, China, between April 2018 and April 2020. The inclusion criteria for CRPC were (a) to abide by the EAU guidelines on CRPC and (b) that patients had available CRPC specimens and complete clinical data. Therefore, 35 CRPC tissues, including frozen and paraffin-embedded tissues, were obtained from the Affiliated Hospital of North Sichuan Medical College (10 cases); the First Affiliated Hospital of Chongqing Medical University, Chongqing, China (18 cases); and the Fuling Central Hospital, Chongqing, China (7 cases). These cases were collected between May 2008 and April 2020. All PCa and CRPC tissues were confirmed by a trained pathologist. The study protocol was approved by the Human Ethics Review Committee of the First Affiliated Hospital of Chongqing Medical University and Ethics Committee of the Affiliated Hospital of North Sichuan Medical College. This study conforms to the provisions of the Declaration of Helsinki. Informed consent was obtained from the patients or their family members prior to inclusion in the study.

### 2.2. Immunohistochemistry

Samples were embedded in formalin and paraffin and cut into 5 *μ*m thick sections. The immunoreactivities of SOX8, Notch4, and Hes5 were investigated by using immunoperoxidase staining (anti-SOX8, 1 : 200, Abcam, cat. no. ab221053; anti-Notch4, 1 : 200, Abcam, cat. no. ab199295). According to staining intensity, samples were scored as follows: 0, no staining; 1, weak staining; 2, light staining; 3, moderate staining; and 4, strong staining. Staining scores ≤ 1 were deemed as a negative expression, and staining scores ≥ 2 were considered positive.

### 2.3. Cell Culture, Treatment, and Transfection

The cell lines RWPE-1, LNCaP, and DU145 were cultured in RPMI-1640 plus 10% fetal bovine serum (FBS) (Gibco-Life, USA) and were maintained in a 5% CO_2_ incubator at 37°C. To construct enzalutamide-resistant cells (Enza-R), LNCaP cells were treated with gradually increasing doses (1 *μ*M, 3 *μ*M, 5 *μ*M, and 10 *μ*M) of enzalutamide (Selleck, USA) up to 10 *μ*M and maintained for at least 6 months [28]. Lentiviruses (Shanghai Gene Pharma Company, China), containing LV-shNC or LV-shSOX8, and LV-NC or LV-SOX8 were added to the culture medium for 8 hours. Enza-R cells were treated with 1 *μ*g/ml puromycin and incubated for 72 hours to generate SOX8-silenced and SOX8-overexpressed stable enzalutamide-resistance cells, respectively. The prostate cancer cell strains were transfected with Ad-SOX8 or Ad-GFP (Shanghai Gene Pharma Company, China), respectively. After 72 h of incubation, follow-up experiments were performed.

### 2.4. Cell Viability by CCK8 Assay

2,000 cells/well were plated into 96-well plates. 10 *μ*l CCK-8 reagents (Solarbio, Beijing, China) were added into each well and incubated for 1 hour, after which the optical density at 450 nm was measured using a microplate reader (Bio-Rad Laboratories, CA, USA). For half maximal inhibitory concentration (IC_50_) of enzalutamide, LNCaP, Enza-R, and DU145 cells were plated into 96-well plates after pretreatment with various agents, such as LV-NC and LV-shSOX8. After 12 hours, these cells were cultured with various concentration enzalutamide (0, 1, 5, 25, 50, 100, 200, 300, and 400 *μ*M) for 48 hours. Optical density was detected at 450 nm using a microplate reader.

### 2.5. Protein Expression by Western Blotting

Total protein was extracted from cell lines using RIPA buffer containing phosphatase inhibitors (Beyotime Institute of Biotechnology, Beijing, China) according to the manufacturer's procedures. Protein samples (50 *μ*g) were transferred to PVDF membranes (EMD Millipore, MA, USA). After blocking with 5% nonfat milk for 2 hours at room temperature, membranes were treated with the following various primary antibodies overnight at 4°C (Table 1). GAPDH was used as a loading control. All Western blot experiments were repeated at least 3 times.

### 2.6. Immunofluorescence

Cells cultured with various treatments were seeded into a 12-well plate and incubated for 24 hours. After fixing with 4% paraformaldehyde for 15 minutes, cells were incubated with various primary antibodies as follows: anti-Notch4, 1 : 100; anti-SOX8, 1 : 200; anti-Notch1, 1 : 100; anti-Hes1, 1 : 100; anti-Hes5, 1 : 150; anti-BCL-2, 1 : 200; and anti-BAX, 1 : 200. Then, the cells were incubated with appropriate secondary antibodies (Zhongshan Golden Bridge Biotechnology, Beijing, China) for 1 hour in the dark room. DAPI (Zhongshan Golden Bridge Biotechnology) was added for nuclear staining.

### 2.7. mRNA Expression by Reverse Transcription-Quantitative PCR (RT-qPCR)

Total RNA was extracted from cells cultured with various treatments through TRIzol and reversed into cDNA using a PrimeScript™ RT reagent kit (Takara, Dalian, China). Primer sequences were as follows: SOX8, sense, 5′-CGAGAGAA-GACGCCTGCT-3′, antisense, 5′-CGTGTTGGAGAATGAGGG-3′; Notch1, sense, 5′GAACGGGGCUAACAAAGAUTT-3′, antisense, 5′-AUCUUUGUUAGCCCCGUUCTT3′; Notch4, sense, 5′-GGAGACT-GCAGACCAGAAGG-3′, antisense, 5′-GACCCTCAGAGTCAGGGAC-A-3′; Hes1, sense, 5′-GGACTAGTATGCCAGCTGATATAATGGAG-3′, antisense, 5′-GAAGATCTAGGTGGGCTAGGGACTTTAC-3′; and Hes5, sense, 5′-GGAATTCCAATGGCCCCCAGCACTGTG-3′, antisense, 5′-GGGTACCCCACGGCCACAGTGCTGG-3′. All RT-qPCR experiments were performed at least 3 times.

### 2.8. Colony Formation Assay

A total of 400 cells/well were plated into 6-well plates and were cultured for two weeks until the number of each clone reached 50 cells. Then, the cells were fixed with 4% paraformaldehyde for 15 minutes and stained with 0.05% crystal violet for 20 minutes at room temperature. Each group was replicated in three wells.

### 2.9. Transwell and Wound Healing Assay

For the Transwell assay, 1.0 × 10^4^ cells were seeded in the upper chamber of the insert with Matrigel (BD Biosciences, USA). After incubation with serum-free medium for 48 h, cells were stained with 0.1% crystal violet and 4% formaldehyde. The number of cells fixed on the bottom membrane of the inserts was counted under an optical microscope. For the wound healing assay, 5 × 10^4^ cells/well were plated into a 6-well plate. After incubating for 24 hours, cells were wounded with a yellow pipette tip. Then, the cells were cultured for 24 hours, and the wound healing was observed under an optical microscope at indicated time-points.

### 2.10. Xenograft and Bone Metastasis Model

Animal studies were performed according to the Institutional Animal Care and Use Committee of Chongqing Medical University. Enza-R cells (3 × 10^8^) infected with LV-NC or LV-shSOX8 were injected subcutaneously into the right flank or the left tibia of surgically castrated nude mice. After two weeks, mice were treated with enzalutamide and RO0429097 by intraperitoneal injection twice per week. The growth of xenograft tumors in the left flank was evaluated and recorded every 5 days. The xenograft tumors in the right flank were harvested after four weeks, while the xenograft tumors in the left tibia were harvested after eight weeks. Bone destruction in the left tibia was observed by X-ray every four weeks. Tumor volume (mm^3^) was calculated as volume (mm^3^) = 1/2 × length × width [2].

### 2.11. Statistical Analysis

Statistical analyses were performed using the SPSS 19.0 software. Numerical data are shown as mean ± SD. Studentʼs *t*-test, *χ*^2^ test, Mann–Whitney test, Pearsonʼs analysis, one-way ANOVA, two-way ANOVA, and Kaplan-Meier survival analysis were performed as appropriate. *P* < 0.05 was used to infer statistical differences.

## 3. Results

### 3.1. SOX8 and Notch Signaling Proteins Are Upregulated in CRPC Tissues

The expression of SOX8, Notch4, and Hes5 was investigated using immunohistochemistry (IHC). The expression of SOX8 in CRPC samples (26/35, 74%) was obviously higher than that found in PCa tissues (19/45, 42%) (Figures 1(a) and 1(d) and Table 2). Similarly, Notch4 and Hes5 were also upregulated in CRPC tissues compared to those of PCa tissues (Figures 1(b), 1(c), 1(e), and 1(f) and Table 2). Furthermore, the expression of SOX8 was positively correlated with Notch4 (*r* = 0.34, *P* = 0.045) and Hes5 (*r* = 0.35, *P* = 0.039) levels (Figures 1(g) and 1(h)). Moreover, as shown in Table 2, PSA was significantly increased in SOX8-positive PCa patients when compared to SOX8-negative patients. Similarly, increased PSA was also found in Notch4-positive and Hes5-positive patients. More importantly, the expression of SOX8 in PCa tissues was positively associated with bone metastatic lesions (*P* = 0.014); this phenomenon was also found in CRPC patients (*P* = 0.001). In addition, Notch4- and Hes5-positive samples (in both PCa and CRPC patients) were also correlated with metastatic lesions of bones. Our findings suggest that a high expression of SOX8, Notch4, and Hes5 could lead to tumor metastasis (Table 2).

Next, a Kaplan-Meier survival analysis was used to evaluate the relationship between the progression-free survival (PFS) of CRPC patients and the expression of SOX8, Notch4, and Hes5. This analysis revealed that the median PFS was 24 months in CRPC patients that were positive for SOX8 and 43 months in SOX8-negative patients (Figure 1(i), *P* = 0.0365). Moreover, the PFS of Notch4-positive CRPC patients was obviously shorter than that of Notch4-negative patients (24 months vs. 50.5 months, *P* = 0.0101) (Figure 1(j)). Finally, the PFS of Hes5-positive CRPC patients was shorter than that of Hes5-negative patients (22 months vs. 38 months, *P* = 0.0235) (Figure 1(k)).

### 3.2. SOX8, Notch4, and Hes5 Are Upregulated in CRPC Cells

To determine a possible role of SOX8 and Notch signaling in CRPC, we constructed Enza-R cells by continuously treating LNCaP with enzalutamide for at least 6 months. As shown in Figure 2(a), the resistance to enzalutamide in Enza-R cells increased nearly 100-fold compared to their parental cells. Next, the expression of SOX8, Notch4, and Hes5 was detected by RT-qPCR, Western blot, and immunofluorescence. As expected, both mRNA and protein expressions of SOX8, Notch4, and Hes5 were upregulated in DU145 and Enza-R cells. However, these proteins were not detected in RWPE-1 cells, while they were weakly detected in LNCap cells (Figures 2(b) and 2(c)). SOX8, Notch4, and Hes5 were also detected in DU145, which were androgen-independent cells (Figures 2(b)–2(d)). These data suggest that upregulation of SOX8 and Notch signaling molecules may play an important role in the development of enzalutamide resistance in CRPC cells.

### 3.3. SOX8 Knockdown Suppresses the Proliferation, Invasion, and Migration of Enza-R Cells

To explore the possible role of SOX8 in malignant biological behaviors of Enza-R cells, this protein was knocked down using lentivirus. The CCK8 assay showed that SOX8 knockdown inhibited the proliferation of both Enza-R and DU145 cells (Figures 3(a) and 3(b)). A colony assay revealed similar results (Figures 3(c) and 3(d)). To explore the role of SOX8 in invasion and migration of DU145 and Enza-R cells, epithelial-mesenchymal transition (EMT) proteins, such as E-cadherin, N-cadherin, Vimentin, and Zeb-1, were detected by Western blot. It was evident that SOX8 knockdown was associated with the upregulation of E-cadherin and the downregulation of N-cadherin, Vimentin, and Zeb-1, indicating that SOX8 potentiates the metastatic capacity of CRPC cells (Figure 3(e)). Similarly, as shown in Figures 3(f)–3(i), knocking down SOX8 significantly inhibited the invasion and migration of DU145 and Enza-R cells. Surprisingly, knocking down SOX8 reduced enzalutamide resistance by 4-fold, indicating that SOX8 is key to enzalutamide resistance (Figure 3(j)).

### 3.4. SOX8 Knockdown Inhibits Malignant Biological Behaviors of Enza-R Cells through Regulating the Notch Signaling Pathway

As mentioned above, the expression of SOX8 was positively correlated with Notch signaling in CRPC tissues (Figures 1(g) and 1(h)). We hypothesized that knocking down SOX8 would inhibit malignant biological behaviors of resistant cells through the downregulation of Notch signaling. As shown in Figures 4(a)–4(d), SOX8 knockdown obviously downregulated the expression of Notch1, Notch4, and their downstream effectors, such as Hes1, Hes5, Hey1, and Hey2 both at the mRNA and protein levels. To determine the role of Notch signaling in Enza-R cells, we treated cells with 5 *μ*M RO04929097 (a *γ*-secretase inhibitor) for 48 h, which inactivates Notch signaling. As shown in Figure 4(d), a combination of SOX8 knockdown and RO04929097 led to a more potent inhibition of the expression of multiple oncogenic pathways, such as p21 and c-myc. In addition, to investigate the correlation between SOX8 and Cyclin family members in Enza-R cells, the expression of Cyclin E1, Cyclin D1, and Cyclin D3 was detected after knocking down SOX8. As shown in Figure 4(e), downregulation of SOX8 decreased the activity of Cyclin family members, suggesting that the dysregulation of SOX8 promotes the proliferation of Enza-R cells. When SOX8 knockdown cells were treated with RO04929097, there was a more obvious decrease of Cyclin family members, indicating that both SOX8 and Notch signaling are involved in regulating the mitosis of Enza-R cells. Moreover, a synergistic effect between SOX8 downregulation and RO04929097 was observed on the apoptosis of Enza-R cells, as evidenced by the upregulation of BAX and BAK and the downregulation of Bcl-2 and Bcl-xl (Figures 4(e) and 4(f)).

Next, we investigated if SOX8-mediated effects on CRPC cells were due to the regulation of the Notch signaling pathway. Notch4 receptor was knocked down by adenoviruses in LNCaP cells that overexpressed SOX8. The CCK8 assay showed that overexpression of SOX8 promoted the proliferation of LNCaP; however, when Notch4 receptor was concomitantly knocked down, the growth of LNCaP was obviously inhibited (Figures 5(a) and 5(b)). Moreover, knocking down Notch4 impaired the invasion ability caused by the overexpression of SOX8 in LNCaP cells (Figure 5(b)). As shown in Figure 5(c), Notch4 knockdown led to a downregulation of the expression of Cyclin E1, Bcl-2, and N-cadherin and an upregulation of the expression of BAK1 and E-cadherin. Our data suggest that knocking down Notch4 could rescue the proliferation and invasion caused by the overexpression of SOX8 in CRPC cells. More importantly, the overexpression of SOX8 increased enzalutamide resistance by 2-fold. However, when knocking down Notch4, such drug resistance was reversed in LNCaP cells (Figure 5(d)). Taken together, data herein presented support that Notch4 downregulation can rescue the proliferation, invasion, metastasis, and drug resistance caused by the overexpression of SOX8 in CRPC cells, thus inhibiting malignant biological behaviors of CRPC cells.

Xie et al. reported that SOX8 confers chemoresistance and stemness properties and mediates EMT in tongue squamous cell carcinoma via bounding to the promoter region of Frizzled-7 (FZD7) and inducing the FZD7-mediated activation of the Wnt/*β*-catenin pathway [32]. Moreover, previous studies revealed that the induction of the Notch ligand/receptor was regulated by *β*-catenin hyperactivation in intestinal tumorigenesis [35–37]. Therefore, we hypothesized that SOX8 regulates Notch signaling through *β*-catenin in CRPC.

As shown in Figure 5(e), SOX8 downregulation decreased the expression of *β*-catenin, *p-β*-catenin, Notch1, and Notch4. However, when Enza-R cells were treated with AZD2858 (a Wnt/*β*-catenin activator), the downregulation of Notch1 and Notch4 was rescued. Similarly, the combination of knocking down SOX8 and treatment with PNU74654 (a Wnt/*β*-catenin inhibitor) led to a stronger inhibition of Notch signaling molecules when compared to that of either treatment alone. Consistent with our hypothesis, the activation of Notch signal mediated by SOX8 is achieved through the regulation of *β*-catenin in Enza-R cells.

### 3.5. Inhibition of the Notch Signaling Pathway by Both Knocking Down SOX8 and *γ*-Secretase Inhibitor (RO04929097) Significantly Reversed the Enzalutamide Resistance

As mentioned above, downregulation of SOX8 inhibited the proliferation, invasion, and migration of Enza-R cells. Thus, we hypothesized that the overexpression of SOX8 was responsible for enzalutamide resistance in Enza-R cells. As expected, the CCK-8 assay showed that the downregulation of SOX8 increased the sensitivity of the Enza-R cells to enzalutamide by 5.2-fold (Figure 6(a)). Similar results were found in DU145 cells, in which there was a 2.26-fold in reversing resistance (Figure 6(c)), suggesting that dysregulation of SOX8 is responsible for enzalutamide resistance. Importantly, a *γ*-secretase inhibitor named RO04929097 was also able to reversed enzalutamide resistance by 5.8-fold in Enza-R cells and by 1.9-fold in DU145 cells (Figures 5(b) and 5(d)), indicating that pharmacological intervention of Notch signaling by RO04929097 may represent a promising therapeutic strategy for CRPC.

Next, to determine the antitumor effect of RO04929097 on the CRPC cell model, the CCK-8 assay was performed to evaluate the proliferation of Enza-R and DU145 cells following treatment with various concentrations of RO04929097 (5, 10, 20, 30, 40, 60, 80, and 100 *μ*M). As shown in Figures 6(e) and 6(f), RO04929097 exerted a dose-dependent and powerful antitumor effect on both Enza-R and DU145 cells, suggesting that inhibition of *γ*-secretase decreased Notch signaling and may become a novel and potent therapy for CRPC.

### 3.6. Combination of Enzalutamide with RO04929097 Displays a Synergic Effect in Blocking the Growth and Bone Metastasis of Enza-R Cells In Vivo

As mentioned above, SOX8 and Notch inhibitor RO04929097 effectively suppressed malignant biological behaviors of Enza-R cells *in vitro*. Next, we evaluated the therapeutic potential of these strategies *in vivo*. Xenograft tumor models were constructed by treating castrated nude mice with a combination of enzalutamide and RO04929097. Compared to the control group, both LV-shSOX8 and RO04929097 groups had significantly decreased volume and weight of their xenograft tumor (Figures 7(a)–7(c) and 7(f)). Of note, when LV-shSOX8 and RO04929097 were combined, the inhibitory effect became stronger (Figures 7(a)–7(c) and 7(f)). Next, we subcutaneously injected Enza-R cells with LV-NC or LV-shSOX8 into the right tibia to construct a bone metastasis model. Mice were treated with enzalutamide and/or RO04929097 injected into the tail vein. X-ray, H&E histology, and IHC were performed to evaluate bone destruction. As expected, SOX8 knockdown as well as RO04929097 obviously reduced the bone metastasis, compared to the control group (Figures 7(d)–7(f)). Moreover, a synergistic effect was detected in preventing bone destruction when SOX8 knockdown and RO04929097 were combined (Figures 7(d)–7(f)).

## 4. Discussion

In healthy organisms, SOX genes regulate cell differentiation, organogenesis, and many other developmental processes [38–41]. However, SOX gene members are frequently dysregulated in various tumors [42, 43]. SOX2 is weakly detected in benign prostate tissues; however, it is highly expressed in PCa tissues, including in CRPC ones. More importantly, SOX2 promotes tumor tumorigenesis and progression. Reduced SOX2 levels were shown to attenuate the proliferation and invasion while increasing the redifferentiation of PCa cells [44, 45]. Meanwhile, SOX4 is also overexpressed in PCa tissues and cell lines, and its upregulation is correlated with a higher Gleason score. Moreover, decreased SOX4 induces death of PCa cells, indicating that SOX4 might be a therapeutic target for PCa [46, 47]. Interestingly, SOX11 was recently reported to act as a tumor suppressor in PCa, since its overexpression suppressed the migration and invasion of PCa cells [48, 49]. In addition, SOX9, also known as a soxE member, was overactivated in PCa cells and its downregulation inhibited tumorsphere formation in androgen-deficient hosts [50]. In our study, we found that SOX8, another soxE member, was highly expressed in both CRPC tissues and Enza-R cells and that SOX8 was associated with a worse prognosis of CRPC patients. Reducing the expression of this enzyme significantly inhibited malignant biological behaviors of Enza-R cells and reversed enzalutamide resistance, suggesting that SOX8 may be a potential target for CRPC therapy.

The Notch receptor members are recognized as an oncogene in various tumors, including PCa. Notch1 was found to be overactivated in PCa, while its inhibition by a *γ*-secretase inhibitor restored enzalutamide function [24, 26, 27, 51]. Also, inhibition of Notch2 activation by GSI-1, another *γ*-secretase inhibitor, decreased the cell survival of prostate cells and promoted their apoptosis [24, 52]. A recent study reported that Notch3 is responsible for PCa-induced bone lesion by activating MMP-3 signaling [53]. Another study revealed that hypoxia triggers the activation of Notch3, which, in turn, sustains the survival and proliferation of PCa cells *in vivo* [54]. Notch4 is involved in the progression of PCa given that Notch4 ablation inhibits PCa growth and EMT via the NF-*κ*B pathway [55]. Here, we discovered that Notch4 is highly expressed in CRPC tissues and associated with a poorer prognosis of CRPC patients. Our previous studies indicate that Notch receptors 1, 2, 3, and 4 have no statistically significant relationship with bone metastasis [20]. However, the present study found that Notch4 instead of Notch1, 2, and 3 was significantly correlated with bone metastasis (data not show). It can be explained that we have added research center and obtained some new samples from it. Moreover, Notch4 reduction, achieved by knocking down SOX8 and/or treatment with RO04929097, significantly inhibited the survival and growth of Enza-R cells and restored enzalutamide sensitivity in Enza-R cells, suggesting that interfering with the Notch/SOX8 axis may be a potential target for the treatment of CRPC.

## 5. Conclusion

Our data indicated that overactivated SOX8, Notch4, and Hes5 predict more susceptibility to bone metastases and shorter PFS in CRPC tissues. Furthermore, the SOX8/Notch4 signaling axis is responsible for enzalutamide resistance, and knocking down SOX8 may be a novel strategy for the treatment of CRPC. Importantly, the pharmacological inhibition of Notch signaling by RO04929097 may be a promising therapeutic strategy for CRPC.

## Figures and Tables

**Figure 1:** The expression of SOX8, Notch4, and Hes5 in samples of prostate cancer (PCa) and castration-resistant prostate cancer (CRPC) and the Kaplan-Meier survival analysis for the progression-free survival (PFS) of 35 patients with CRPC. (a–c) The expression levels of SOX8, Notch4, and Hes5 were detected by immunohistochemistry (×200). (d–f) Average staining scores for SOX8, Notch4, and Hes5 in PCa and CRPC samples. According to staining intensity, samples were divided as follows: 0, no staining; 1, weak staining; 2, light staining; 3, moderate staining; and 4, strong staining. Staining scores ≤ 1 were defined as having a negative expression, while staining scores of ≥2 were defined as having a positive expression. (g, h) The correlation curve between SOX8 staining scores versus Notch4 or Hes5 staining scores in CRPC tissues. (i–k) Kaplan-Meier survival analysis was used to assess the relationship between PFS and the expression of SOX8, Notch4, and Hes5 in patients with CRPC. *P* < 0.05 was considered to be statistically different.

**Figure 2:** Expression of SOX8 and Notch signaling detected in Enza-R cells. (a) Both LNCaP and Enza-R cells were treated with increasing concentrations of enzalutamide for 24 hours, and the IC_50_ was detected by a Cell Counting Kit-8 (CCK-8) assay. (b–d) mRNA and protein expression of SOX8, Notch4, and Hes5 assessed by RT-PCR, Western blot, and immunofluorescence (×200). ^∗^*P* < 0.05 and ^∗∗^*P* < 0.01. ns: no significance.

**Figure 3:** Knocking down SOX8 inhibits malignant biological behaviors of prostate cancer (PCa) cells that are resistant to treatment. (a, b) The viability of DU145 and Enza-R cells was measured by a CCK-8 assay after knocking down SOX8. (c, d) Colony-forming efficiency of DU145 and Enza-R cells after 10 days of culture. (e) The expression of E-cadherin, N-cadherin, Vimentin, and Zeb-1 in both DU145 and Enza-R cells was examined by Western blot. Cells were transfected with lentiviruses containing LV-NC or LV-shSOX8. GAPDH served as a loading control. (f, g) A Transwell assay was performed to examine the invasive ability of DU145 and Enza-R cells following SOX8 knockdown (magnification, ×400). (h, i). The migratory capacity of Enza-R cells was evaluated after the cells were wounded with a yellow pipette tip for 0 h, 24 h, and 48 h. (j) Enza-R cells were exposed to increasing concentrations of enzalutamide (0, 1, 5, 25, 50, 100, 200, 300, and 400 *μ*M) for 48 h, and the half maximal inhibitory concentration (IC_50_) was determined by a CCK8 assay. ^∗^*P* < 0.05 and ^∗∗^*P* < 0.01. Enza-R: enzalutamide-resistant LNCaP cells.

**Figure 4:** Knocking down SOX8 and treatment with RO04929097 inhibit Notch signaling and its downstream. (a–c) Notch signaling activity in Enza-R cells after knocking down SOX8 was detected by RT-qPCR, Western blot, and immunofluorescence. Cell nuclei were stained with DAPI (magnification, ×200). In order for the figure to be more concise, panels for DAPI staining alone are not shown. (d–f) Downstream genes of Notch signaling were detected in DU145 and Enza-R cells after knocking down SOX8 and/or treating with RO04929097 using Western blot and immunofluorescence. ^∗∗∗^*P* < 0.001; GAPDH served as a loading control. Enza-R: enzalutamide-resistant LNCaP cells.

**Figure 5:** Notch4 knockdown rescued the proliferation, invasion, metastasis, and drug resistance caused by the overexpression of SOX8 and SOX8-regulated Notch signaling through *β*-catenin protein. (a) The viability of LNCaP cells was measured by a CCK-8 assay after knocking down Notch4 using adenoviruses in cells that overexpressed SOX8. (b) Colony-forming efficiency of SOX8-overexpressing Notch4 knocked down LNCaP cells after 10 days of culture. The Transwell assay was performed to examine the invasive ability of LNCaP cells following SOX8 overexpression and Notch4 knockdown (magnification, ×400). (c) Cyclin D1, Cyclin E1, BAK1, and Bcl-2 were detected using Western blot assay; GAPDH served as a loading control. (d) LNCaP cells were exposed to increasing concentrations of enzalutamide (0, 0.3, 0.6, 1.2, 2.4, 3.6, 4.8, 6.0, and 7.2 *μ*M) for 48 h, and the half maximal inhibitory concentration (IC_50_) was determined by a CCK-8 assay. (e) Enza-R cell was subjected to SOX8 knockdown and/or treatment with AZD2858 (5 nM 24 hours) or PNU74654 (5 nM 24 hours). The expression of SOX8, *β*-catenin, p-*β*-catenin, Notch1, and Notch4 was detected by Western blot assay; , GAPDH served as a loading control, ^∗∗∗^*P* < 0.001.

**Figure 6:** Knocking down SOX8 and treatment with RO04929097 resensitized Enza-R and DU145 cells to enzalutamide, while RO04929097 exerts an antitumor effect on resistant cells. (a–d) Enza-R and DU145 cells were subjected to SOX8 knockdown and/or treated with RO04929097. Cells were exposed to increasing concentrations of enzalutamide (0, 1, 5, 25, 50, 100, 200, 300, and 400 *μ*M) for 48 h, and the half maximal inhibitory concentration (IC_50_) was determined by a CCK-8 assay. (e, f) Enza-R and DU145 cells were treated with increasing concentrations of PF-3084014 (2, 5, 10, 20, 30, 40, 60, 80, and 100 *μ*M) or DMSO for 48 h. Cell viability was detected by a CCK-8 assay. ^∗∗^*P* < 0.001. Enza-R: enzalutamide-resistant LNCaP cells.

**Figure 7:** Knocking down SOX8 and/or treatment with RO04929097 suppress the growth and bone metastasis of Enza-R cells *in vivo*. Nude mice with subcutaneous or bone xenograft tumors were treated with 10 mg/kg enzalutamide and 50 mg/kg RO04929097. (a) Tumor growth curve. (b) Weight of tumors. (c) Images of the recovered tumors. (d) X-ray of bone metastasis (red arrow). (e) H&E staining of bone metastasis (upper ×100, lower ×200; black arrow). (f) The expression of SOX8 and Notch4 in xenograft and bone lesion was detected by IHC. ^∗^*P* < 0.05; ^∗∗∗^*P* < 0.001; Enza-R: enzalutamide-resistant LNCaP cells.

**Table 1:** Primary antibodies for Western blotting assay.

Primary antibodies	Concentration	Company	Catalog number
SOX8	1 : 2,000	Abcam	ab104245
Notch4	1 : 1,000	Santa Cruz	SC-383993
Hes5	1 : 2,000	Abcam	ab25374
E-Cadherin	1 : 2,000	CST	14472
N-Cadherin	1 : 2,000	CST	13116 s
Vimentin	1 : 1,000	CST	5741 s
Zeb-1	1 : 2,000	CST	70512 s
Hey1	1 : 2,000	Abcam	ab22641
Hey2	1 : 1,000	Abcam	ab167280
P21	1 : 2,000	Abcam	ab109520
c-Myc	1 : 1,000	Abcam	ab32072
Cyclin E1	1 : 1,000	Abcam	ab33911
Cyclin D1	1 : 2,000	Abcam	ab16663
Cyclin D3	1 : 1,000	Abcam	abSP207
BAX	1 : 2,000	Abcam	ab53145
BAK	1 : 2,000	CST	12105T
BCL2	1 : 2,000	CST	4223T
BCL-xl	1 : 1,000	CST	2764T
*β*-Catenin	1 : 1,000	Abcam	ab223075
*p*-*β*-Catenin	1 : 500	Abcam	ab277785
GAPDH	1 : 1,000	CST	5174s

Abcam: Abcam Cambridge, UK; Santa Cruz: Santa Cruz Biotechnology, Inc., USA; CST: Cell Signaling Technology, USA.

**(a):** 

	SOX8 expression in PCa			SOX8 expression in CRPC		
	Negative 26/45 (58%)	Positive 19/45 (42%)	*P* value	Negative 9/35 (26%)	Positive 26/35 (74%)	*P* value
Median of PSA (*μ*g/L)	15.55	27.33	P = 0.039^a^	14.93	23.33	P = 0.37^a^
Quartiles 25-75	11.46-33.20	16.09-41.32		10.36-46.47	12.58-33.84	
Gleason score	*N* = 26	*N* = 19	P = 0.33^b^	N = 9	N = 26	P = 0.24^b^
≤7	13/26 (50%)	12/19 (63%)		3/9 (33%)	10/26 (38%)	
≥8	13/26 (50%)	7/19 (37%)		6/9 (67%)	16/26 (62%)	
(New)bone metastasis	7/26 (27%)	13/19 (68%)	P = 0.014^c^	4/9 (44%)	25/26 (96%)	P = 0.001^c^

**(b):** 

	Notch4 expression in PCa			Notch4 expression in CRPC		
	Negative 23/45 (51%)	Positive 22/45 (49%)	*P* value	Negative 8/35 (22%)	Positive 27/35 (78%)	*P* value
Median of PSA (*μ*g/L)	14.55	25.89	P = 0.022^a^	13.84	23.33	P = 0.16^a^
Quartiles 25-75	10.66-32.56	15.91-65.07		10.36-29.90	12.58-35.73	
Gleason score	N = 23	N = 22	P = 0.42^b^	N = 8	N = 27	P = 0.32^b^
≤7	10/23 (43%)	10/22 (45%)		2/8 (25%)	11/27 (41%)	
≥8	13/23 (57%)	12/22 (55%)		6/8 (75%)	16/27 (59%)	
(New)bone metastasis	6/23 (26%)	14/22 (64%)	P = 0.011^c^	4/8 (50%)	25/27 (93%)	P = 0.006^c^

**(c):** 

	Hes5 expression in PCa			Hes5 expression in CRPC		
	Negative 24/45 (53%)	Positive 21/45 (47%)	*P* value	Negative 11/35 (31%)	Positive 24/35 (69%)	*P* value
Median of PSA (*μ*g/L)	15.96	25.33	P = 0.029^a^	15.31	23.54	P = 0.40^a^
Quartiles 25-75	10.40-31.20	15.70-52.23		11.72-34.23	12.34-35.11	
Gleason score	N = 24	N = 21	P = 0.40^b^	N = 11	N = 24	P = 0.21^b^
≤7	11/24 (46%)	8/21 (38%)		2/11 (18%)	11/24 (46%)	
≥8	13/24 (54%)	13/21 (62%)		9/11 (82%)	13/24 (54%)	
(New)bone metastasis	7/24 (29%)	13/21 (62%)	P = 0.027^c^	7/11 (64%)	22/24 (92%)	P = 0.048^c^

PSA: prostate-specific antigen; PCa: prostate cancer; CRPC: castration-resistant prostate cancer. ^a^Mann-Whitney test. ^b^Chi-square test. ^c^McNemer test. Numbers in italic font indicate statistical significance. *P* < 0.05 was confirmed as statistically significant differences.

## Data Availability

All datasets of this article are included within the article. More supporting data is available under reasonable request.

## Abbreviations

CRPC: Castration-resistant prostate cancer
PCa: Prostate cancer
IHC: Immunohistochemistry
FBS: Fetal bovine serum
CCK-8: Cell Counting Kit-8
Enza-R: Enzalutamide-resistant cells
RIPA: Radio immune-precipitation assay
PVDF: Polyvinylidenefluoride
RT-qPCR: Reverse transcription-quantitative polymerase chain reaction
SPSS: Statistical product and service solutions
PFS: Progression-free survival
EMT: Epithelial-mesenchymal transition
FZD7: Frizzled-7
H&E: Hematoxylin-eosins.
